# A Two-Year Longitudinal Study of the Effectiveness of the CRT^®^ Bacteria Test in Evaluating Caries Risk in Three-Year-Old Children

**DOI:** 10.1155/2021/7488855

**Published:** 2021-10-05

**Authors:** Yun Liu, Yusheng Meng, Min Wu, Qian Zhang

**Affiliations:** Stomatological Healthcare Center, Shenzhen Maternity and Child Healthcare Hospital Affiliated to Southern Medical University, Shenzhen 518048, China

## Abstract

**Objective:**

To study the correlation between the level of infection with *Streptococcus mutans* (SM) and lactobacilli (LB) in saliva with existing status and the development of primary dental caries in 3-year-old children and to evaluate the results of CRT^®^ bacteria as a Caries Risk Test.

**Methods:**

A total of 140 3-year-old children were selected for the study. Oral examination was conducted and the levels of infection with SM and LB in saliva were measured using a CRT^®^ bacteria test. Oral reexamination was conducted after two years. The prevalence rate of caries, the decayed-missing-filled tooth (dmft) and decayed-missing-filled surface (dmfs) indices, and Caries Severity Index (CSI) were calculated at the start and end of the two years. The indices were statistically analyzed.

**Results:**

The caries prevalence rate, dmft, dmfs, and CSI increased with increasing levels of CRT-SM and CRT-LB at the start and end of the two years; the increases in dmft, dmfs, and CSI over the period were consistent with the increases in CRT-SM and CRT-LB levels, with all differences being highly statistically significant. The increase in caries prevalence rate over the two years was not statistically different for different CRT-SM and CRT-LB levels. CRT-SM and CRT-LB levels were highly positively correlated with dmft, dmfs, CSI and their increases over the two years. Levels of infection with oral SM and LB were found to be independent risk factors for primary dental caries, respectively. For an SM concentration in saliva of ≥10^4^ CFU/mL and an LB concentration of <10^4^ CFU/mL, the risk of caries increased by approximately 2.8-fold. When the concentration of LB in saliva was ≥10^4^ CFU/mL and that of SM <10^4^ CFU/mL, the risk of caries increased by approximately 3.9-fold. When the concentration of both SM and LB was ≥10^4^ CFU/mL, the risk increased by approximately 10.9-fold.

**Conclusions:**

Significant positive correlations were found between the level of infection with oral SM and LB and existing oral decay status and the trend in the development of primary dental caries. Infection with SM and LB significantly increased the risk of caries in primary teeth. The CRT^®^ bacteria is a simple, convenient, reliable, and effective Caries Risk Test.

## 1. Introduction

The most common chronic illness among children globally in both developed and developing countries is caries [1, 2]. The prevalence of childhood caries remains the highest of all childhood diseases, five times greater than that of asthma and seven times that of hay fever [1]. Untreated primary dental caries affected 621 million children worldwide in 2010, representing approximately 9% of the global population [2]. In 2005 and 2015, the 3^rd^ and 4^th^ national oral epidemiological surveys were conducted in China, and the results revealed that the prevalence rate of caries and the mean value of the decayed-missing-filled tooth (dmft) index in 5-year-old children were 66.0% and 3.5 in 2005 and 71.9% and 4.24 in 2015, respectively, reflecting a significant deterioration in oral health [3, 4]. The 3^rd^ oral epidemiological survey in China found that 79.3% of caries in children aged 5 years was concentrated in one-third of the population with a mean dmft value of 8.33, and the 4^th^ survey reported that 75.4% of caries in 5-year-old children could be found in one-third of the population with a mean dmft value of 9.61 [4]. An oral epidemiological survey conducted in the US also found that 20% of the population suffered from approximately 60% of all caries [5]. Evidence indicates a skewed distribution of caries in the population, with a particular subpopulation susceptible to severe caries [3–5].

Caries are a chronic infectious illness resulting from the interaction of multiple factors, such as varying microorganisms, the host, and dietary factors [6, 7]. A wide range of bacteria grow in the oral cavity and the population undergoes pathological evolution and change during the development of caries in children, from an equilibrium state with multiple bacteria to one in which a few cariogenic bacteria predominate [7–9]. Furthermore, cariogenic bacteria decompose and ferment food to produce acid which gradually erodes the teeth, eventually leading to demineralization and so caries [6]. In particular, *Streptococcus mutans* (SM) and lactobacilli (LB) are considered the primary cariogenic bacteria [6, 9].

Caries risk refers to the sensitivity of a host to caries, reflecting their susceptibility and propensity to develop caries [6]. A Caries Risk Test (CRT) aims to detect risk factors for the occurrence of caries by objectively evaluating the risk of caries or the level of caries activity in an individual which is significant for the prevention and control of caries in high-risk populations [6].

In the present study, we conducted an investigation of 3-year-old children from the Shenzhen Kindergarten, Guangdong Province, China, in which oral examinations were performed and tests for levels of infection with SM and LB in saliva using a CRT^®^ bacteria test, from which the correlation between the level of SM and LB infection and the development and status of primary dental caries was calculated, as well as the ability of the CRT^®^ bacteria test to function as a CRT during surveillance of the occurrence and development of caries in children.

## 2. Materials and Method

### 2.1. Subjects

The present study was approved by the Medical Ethics Committee of Shenzhen Maternity and Child Healthcare Hospital (Clinical Trial Registration Number: [2018]106). 3-year-old children in Shenzhen Kindergarten were recruited to the study and followed up for two years. The inclusion criteria for participants were as follows:

- Healthy children with no systemic disease, 3 years of age at the time of screening
- Willing to accept oral examination and collection of a saliva sample stimulated using paraffin
- No antibiotics use for two weeks prior to saliva collection
- No professional fluoride treatment within the 48 hours prior to saliva collection
- No use of an antimicrobial mouth rinse for 12 hours prior to saliva collection
- Signed parental consent or that of a legal guardian or a family member that is the primary care provider when the primary caregiver is not the parent

The results of the first clinical examination and reexamination after two years were provided to the parents in written form. Parents were provided oral healthcare guidance each year, principally relating to the children's diet, and oral cleaning and healthcare, such as the impact of sugar consumption and the frequency of its consumption on oral health, the need to gargle after eating, the use of fluoride toothpaste, teaching parents how to brush and floss for children, and the importance of regular oral examination.

### 2.2. Research Method

Oral examination and the relative measurement of SM and LB infection levels in saliva were conducted for each individual at the initial clinical examination. Only an oral examination was conducted at the clinical reexamination after two years.

#### 2.2.1. Oral Examination

The initial and follow-up oral examinations were conducted by the same senior pediatric dentist. The kappa statistic was calculated for both examinations, the resultant values were found to be greater than 0.9, indicating that the results were reliable [10, 11].

The dentist performed a diagnosis both visually in natural light and with probing using a disposable mirror and probe, with all examination results recorded contemporaneously.

The diagnostic criteria of caries as described in the *Oral Health Surveys: Basic Methods* by the World Health Organization (WHO) [12] was used, any uncertain cases being excluded. The type of caries was also recorded, such as secondary caries, enamel caries, dentin caries, or that of the residual crown or residual root.

#### 2.2.2. Indicators of Caries Status

Based on the oral examination results, the prevalence rate of caries, dmft, decayed-missing-filled surface (dmfs), and Caries Severity Index (CSI) were calculated [6, 13]. CSI was scored using the caries criteria developed by Shimono et al. [13]: 0 if a tooth was sound; 0.5 where a filling was present; 1 if secondary caries was present after the filling had been placed, enamel caries, or superficial dentin caries; and 2 when deep caries of the dentin was present, or exposure of the endodontium, or a residual crown, or root was observed. The highest score was recorded if multiple decayed surfaces were detected on one tooth.

  Caries prevalence rate = (number of cases of caries/total number of participants) × 100%.
  dmft = numbers of decayed teeth (dt) + missing teeth (mt) + filled teeth (ft).
  dmfs = numbers of decayed surfaces (ds) + missing surfaces (ms) + filled surfaces (fs).
  CSI = [sum of caries scores ÷ (number of teeth × 2)] × 100.

#### 2.2.3. Measurement of Levels of Infection of Oral SM and LB

A standard CRT^®^ bacteria kit (Ivoclar Vivadent Inc., Liechtenstein) was adopted in the present study, containing paraffin pellets and two special plates. One side of the special plate was covered with black SM selective culture medium (MSB) and the other side coated with green LB selective culture medium (Rogosa Agar). The test was performed between 9 and 10 a.m. Participants fasted for one hour prior to the examination. The specific collection procedure was as follows: stimulated saliva was obtained from the children by asking them to chew the paraffin pellets prior to its collection in a sterile sputum cup. The agar was entirely covered with saliva. The carrier was then held slightly obliquely to allow excess saliva to flow out. The agar was held upright and placed tightly to form a seal. No contact by the researcher was permitted with the surface of agar during the entire process. The agar plates were incubated at 37°C for 48 h and the colony density of SM and LB was recorded. The numbers of SM and LB on the agar were compared with a standard plate and the results recorded accordingly.

Numbers of CRT-SM and CRT-LB observed were categorized into the following levels: level 0: bacterial count <10^4^ CFU/mL; level 1:10^4^ CFU/mL ≤ bacterial count <10^5^ CFU/mL; level 2: 10^5^ CFU/mL ≤ bacterial count <10^6^ CFU/mL; and level 3: bacterial count ≥10^6^ CFU/mL.

### 2.3. Sample Size

This was a prospective cohort study. From the data in a previous report [14], the two-year increment for decayed-filled surface (dfs) of CRT-SM at levels 0, 1, 2, and 3 were 1.53 ± 2.43, 2.75 ± 3.12, 6.91 ± 6.49, and 9.61 ± 6.19, and CRT-LB at levels 0, 1, 2, and 3 were 1.54 ± 3.21, 3.80 ± 4.82, 6.82 ± 4.83, and 10.36 ± 7.52, respectively. For a two-sided test where *α* = 0.05 and *β* = 0.10 with power = 90%, the sample size N for a study of SM was 64 cases, and 80 cases for a study of LB, as calculated using PASS 15 software. Considering a loss to follow-up of 15%, at least 92 cases should be included.

In the present study, all the 3-year-old children in the same kindergarten in Shenzhen were selected. A total of 143 3-year-old children were included in the first clinical examination. After two years, 3 children had withdrawn from the kindergarten due to the family moving away, a rate of loss in the follow-up of 2.10%. A total of 140 children completed the two-year follow-up, half male and half female.

### 2.4. Statistical Analysis

A normality test, Chi-square test, Kruskal–Wallis test, Wilcoxon signed-rank test, and logistic regression with Spearman's rank correlation coefficient were calculated in the present study. All statistical analyses were conducted using SAS 8.02 software. The results of two-sided tests were considered statistically significant where *P* < 0.05 and highly significant at *P* < 0.01.

## 3. Results

### 3.1. Oral Examinations for Caries

In the initial oral examination, the prevalence of caries in the 140 children was 34.29%, with dmft, dmfs, and CSI values of 1.48, 2.23, and 4.71, respectively. In the follow-up oral examination two years later, the prevalence was 66.43%, and the values of dmft, dmfs, and CSI were 3.81, 6.08, and 11.87, respectively. No significant difference between the genders in the indicators of caries status at the initial exam and after two years was observed, nor an increase in indicator values over the two years (Table 1).

### 3.2. Correlation between the Caries Status and CRT-SM Levels

Table 2 displays the caries status and statistical analysis of the two oral examinations of the 140 children at each CRT-SM level. The prevalence of caries, dmft, dmfs, and CSI at each CRT-SM level at both the initial and the follow-up examinations and the increase in dmft, dmfs, and CSI over the two years increased with increasing CRT-SM level, at high levels of statistical significance. The prevalence of caries, dmft, dmfs, and CSI was statistically different when comparing CRT-SM levels 0, 2, and 3 at the initial oral examination. At the follow-up examination, the prevalence of caries was statistically different between CRT-SM levels 0 and 3, in addition to between levels 1 and 3, and dmft, dmfs, and CSI were statistically different between CRT-SM levels 0, 2, and 3, between levels 1 and 3, and between levels 2 and 3. The increase in dmft, dmfs, and CSI during the two years was found to be statistically different between CRT-SM level 3 and all other levels. No statistical difference was found for the increase over two years of caries prevalence rate between each CRT-SM level.

Table 3 displays the results of statistical and correlation analysis between the CRT-SM levels and indicators of caries status, such as dmft, dmfs, and CSI in the two oral examinations and the increase in values of indicators over the two years. All were positive correlations with coefficients ranging from 0.30 to 0.41 (*P* < 0.01).

### 3.3. Correlation between Caries Status and CRT-LB Levels

Statistical analysis of caries status at each CRT-LB level of the two oral examinations of the 140 children is presented in Table 4. The prevalence of caries, dmft, dmfs, and CSI increased with increased CRT-LB level at both the initial and follow-up examinations, with dmft, dmfs, and CSI increasing over the two years with increased CRT-LB level, at a high level of statistical significance. In the initial oral examination, the prevalence of caries was significantly different between CRT-LB level 0 and all other levels, and dmft, dmfs, and CSI were statistically different between CRT-LB levels 0, 2, and 3. In the follow-up examination after two years, the prevalence was statistically different between CRT-LB levels 0 and 2, with dmft, dmfs, and CSI significantly different between CRT-LB levels 0, 2, and 3, and levels 1, 2, and 3. The increase in dmft and dmfs over the two years was statistically different between CRT-LB levels 0 and 2, with CSI significantly different between CRT-LB levels 0, 2, and 3, and between levels 1 and 2.

Table 5 displays the results of statistical and correlation analysis between CRT-LB levels and the indicators of caries status, such as dmft, dmfs, and CSI in the two examinations and the increase in values of indicators over the two years, all positively correlated with coefficients ranging from 0.26 to 0.39 (*P* < 0.01).

### 3.4. Logistic Regression Model for Caries Status at Different Levels of Infection with Cariogenic Bacteria

#### 3.4.1. Single-Factor Logistic Regression Model for Caries Status at Different Levels of Infection with Cariogenic Bacteria

The single-factor logistic regression analysis of the impact of various levels of infection with oral cariogenic bacteria on caries status is displayed in Table 6, suggesting that both SM and LB infections are independent risk factors for caries in primary teeth.

#### 3.4.2. Multivariate Logistic Regression Model for Caries Status at Different Levels of Infection with Cariogenic Bacteria

The results of multivariate logistic regression analysis of the impact of different levels of infection of oral SM and LB on caries status found *χ*^2^ = 19.9783 with *P* < 0.0001, a highly significant result (Table 7). The parameters obtained and the statistical analysis are shown in Table 8. Furthermore, the resultant probability of caries was calculated to be *p* = Pr (caries = 1) = e^−2.2740+1.0442∗^^SM+1.3482∗^^LB^/(1 + e^−2.2740+1.0442∗^^SM+1.3482∗^^LB^), with the odds of caries increasing 2.8-fold when SM ≥ 10^4^ CFU/mL and LB < 10^4^ CFU/mL in saliva, 3.9-fold when LB ≥ 10^4^ CFU/mL and SM < 10^4^ CFU/mL in saliva, and 10.9-fold when both SM and LB were equal to or greater than 10^4^ CFU/mL.

## 4. Discussion

Both SM and LB are naturally present within the human oral microbiota [6–8]. SM is a chain-like coccus 0.5∼0.8 *μ*m in length and can be observed everywhere in the human mouth [15]. LB is rod-shaped bacteria, not generally abundant in the oral cavity, accounting for approximately 1% of the total salivary flora, and can often be obtained from the surface of the tongue, oral saliva, and decayed teeth [16–18]. SM and LB share the following biological characteristics: they are Gram-positive; they are acidogenic and aciduric bacteria that can survive in a strongly acidic environment and continue to ferment sugars to produce lactic acid; they rely on glycolysis for energy; and they are microaerophiles and require similar nutrition [18, 19]. Hence, both SM and LB can survive and thrive in low pH in addition to environments with inadequate oxygen or nutrition [18, 19]. Furthermore, SM-derived glucosyltransferase can synthesize glucans by fermenting sucrose [20, 21]. Glucan is a high-molecular weight polymer that can be both water-soluble and water-insoluble. Soluble glucan can act as a reserve source of energy, while insoluble glucan is highly viscous and plays an important role in SM adhesion and aggregation to the surface of teeth [20, 21]. Additionally, surface proteins on SM are also important factors for adhesion, which can selectively attach the bacteria to the surface of tooth enamel to form dental plaque [20, 22]. Unlike SM, LB have no adherent surface proteins because they do not produce large quantities of extracellular polysaccharides to promote adhesion, and therefore have a low affinity for dental tissue, thereby often presenting at low levels in plaques [16].

A clinical study investigating changes in the proportion of cariogenic bacteria in dental plaques during the development of caries in children's primary teeth indicated that the percentage of SM in a complete plaque was 16.35%, 26.10%, and 37.24% in precaries, enamel caries, and superficial dentin caries, respectively, and the proportion of LB was extremely low, 0.02%, and 7.17% in precaries, enamel caries, and superficial dentin caries, respectively. The increase in both SM and LB was statistically significant, indicating that SM was the primary cariogenic bacteria and that LB was not the initiating factor in the development of caries but the driving factor in its progression [23].

In the results of the present study, the prevalence of caries, dmft, dmfs, and CSI significantly increased with the increasing CRT-SM and CRT-LB levels at both the initial and follow-up examinations (*P* < 0.01), suggesting that the children with different levels of infection of oral SM and LB had significant differences in caries status, with caries severity increasing as concentration levels of SM and LB increased in the saliva. In children with different levels of CRT-SM and CRT-LB, although there was no statistical difference in the increase in caries prevalence over two years, the increase in dmft, dmfs, and CSI over the two years was highly significant (*P* < 0.01). Increasing evidence has emphasized the contribution of SM and LB to caries. Beighton et al. [24] demonstrated that SM and LB are detected in children with caries significantly more frequently than in caries-free children. Lin et al. [25] studied children aged 3 to 4 years and found that, in the caries group with mean dmft of 9.00 and caries-free group, SM was present in 95.0% and 65.0% of cases, respectively, and LB in 42.5% and 10.0%, respectively, differences that were significant in each case. Matee et al. [26] discovered that the mean SM and LB counts in dental plaque in children with rampant caries were 100-fold higher than in caries-free children, indicating that the level of infection with salivary SM is directly related to rampant caries status. Mattos-Graner et al. [27] studied children aged 1 to 2.5 years and established that children with high levels of infection of salivary SM had a higher prevalence of caries than those with low infection levels. Additionally, Wu et al. [28] observed 8-month-old infants and conducted caries and LB tests in their plaque every 6 months until 32 months of age, revealing that measurements of LB were significantly higher in all age groups than in caries-free infants.

The levels of CRT-SM and CRT-LB were highly positively correlated with dmft, dmfs, and CSI in the two oral examinations and their increase over the two years, further demonstrating that the levels of infection of oral SM and LB are associated with the severity and activity of caries in children [6]. SM and LB can colonize the mouth in early infancy [26]. Teanpaisan et al. [29] conducted a longitudinal study of 169 infants aged 3 to 24 months and found that the detection rates of SM and LB in the saliva of 3-month-olds were 1.78% and 8.88%, respectively, and 86.98% and 66.86% by 24-months, respectively. Moreover, the detection rate of LB in children aged 3–9 months was evidently higher than that of SM, and the rate of SM in children aged 18–24 months was considerably higher than that of LB [29]. The risk of caries in children aged 12–24 months with an SM count >50 CFU/1.5 cm^2^ in the saliva was found to be 7.5–13.0-fold higher than in children without SM infection, and the risk of caries was 3.1- and 13.3-fold higher in children aged 24 months with salivary LB counts of 1–50 and >50 CFU/1.5 cm^2^, respectively, compared with children without LB infection. Importantly, children in whom SM and LB had colonized the oral cavity at early time point were more susceptible to caries, the level of infection with SM and LB positively correlated with the caries status of the children [29]. Kanasi et al. [30] also reported that the level of infection with oral SM and LB was positively correlated with caries in children, and a risk marker for early childhood caries. The results of the present study confirmed that infection with SM and LB are independent risk factors for caries in primary teeth, with the risk of caries increasing approximately 10.9-fold when both SM and LB counts are ≥10^4^ CFU/mL in saliva. Li et al. [31] researched 3- and 5-year-old children and found that the risk of caries increased 6-8-fold when SM were present at >10^6^ CFU/mL in saliva. Hong et al. [32] investigated the association between the concentration of salivary SM in children aged 11 to 12 years and caries; their findings demonstrate that the concentration of salivary SM in children with caries was significantly higher than that of caries-free children, with a highly positive correlation between the concentration of SM in saliva and caries. Moreover, Hong and Hu [32] also concluded that the prevalence of caries in children increases exponentially at an SM concentration of 8.64 × 10^7^/L in saliva.

High levels of infection with SM and LB in childhood caries and their capacity to generate a low pH environment, in addition to their pathogenicity and aciduric properties, indicate that they are key determinants of the development and progression of caries [16]. In the present study, we found that the level of infection of oral SM and LB reflects the caries status and its progression in primary teeth, while a high concentration of SM and LB in saliva predicts an increasing trend for caries in the future. Matee et al. [26] pointed out that there is no difference in SM count in dental plaque and healthy enamel surfaces, but the LB count in dental plaque is 100-fold higher than on a healthy tooth surface, and the proliferation of LB in caries lesions suggests that LB is associated with the progression and severity of caries. Studies have revealed that SM is the bacteria that is cariogenic rather than LB, whereas LB is involved in the development of caries. Specifically, LB counts gradually increase in dental plaque after caries has occurred in normal plaque, lowering the pH and thus affecting the development of caries [17, 18]. It has also been concluded that LB and SM interact and operate in combination during the development and progression of caries. LB is an indirect indicator of fermentable carbohydrate [16, 18].

Caries is a chronic infectious disease that is affected by multiple factors. In addition to microbiological factors, children's feeding and oral hygiene habits are also closely related to the occurrence and development of caries [6, 7]. Studies have demonstrated that the risk factors for caries in young children are a delay to start to brush their teeth, the absence of toothpaste, a high frequency of sweets, and their frequent consumption [6, 33]. All subjects in the present study were from the same kindergarten in Shenzhen. The composition of the diet and the frequency of its consumption in the kindergarten were identical for each child. The children were from civil servants' families living close to the kindergarten, with relatively little mobility. The parents that had been provided with oral healthcare guidance every year were relatively consistent in how they had educated their children and the habits they had retained, reducing the impact of host and dietary factors on the research results to the greatest extent, although this was also a limitation of the study. The caries diagnostic criteria as described in the *Oral Health Surveys: Basic Methods (5th Edition)* formulated by the WHO [12] in 2013 were used in the present study. Caries with cavitated lesions were examined and recorded, but early caries of the enamel with initial noncavitated lesions were not observed and evaluated, a limitation of the WHO caries diagnostic criteria and also the present study. In addition, if follow-up observation data a year after initial examination and additional follow-up examinations over a longer duration had been available, such as three years, the research results would be more complete and the data more convincing.

A Caries Risk Test contributes to the identification of populations with high caries activity or at high risk of causing caries [6]. An ideal Caries Risk Test has the following attributes: consistency with clinical findings; high reproducibility; the ability to reflect current caries status and predict caries trends; ease of use; short test duration with high accuracy; and the capacity to present individual characteristics [34]. At present, no Caries Risk Test fully meets the aforementioned criteria [34]. Tests often require sampling from dental plaque, saliva, and teeth [25–28, 35–37]. Saliva is a bridge between different tissues and structures in the oral cavity and serves as an oral microecological medium with a large number of microorganisms that remain relatively stable [36]. The collection of saliva is a simple, noninvasive, and acceptable approach and a common source for oral clinical research [18, 32, 36]. Evidence has shown that a dynamic balance exists between the bacteria in saliva and dental plaque, with SM and LB counts in saliva highly correlated with the number of corresponding cariogenic bacteria in dental plaque [18]. Motisuki et al. [36] compared the influence of different sample types and collection methods on SM and LB counts and found that the number of SM identified in whole saliva and in dental plaque were similar, whereas the number of LB detected using a whole saliva method was superior to the dental plaque method, suggesting that whole saliva is sensitive to LB measurements. The present study utilized stimulated whole saliva as the sample collected from 3-year old children, who showed a high level of cooperation. The results of the study demonstrated that levels of infection with SM and LB in saliva can be used to predict caries risk in children [37–41].

In the present study, we leveraged the CRT^®^ bacteria test for semiquantitative measurement of SM and LB in saliva; the results showed that the test represents a simple, convenient, reliable, and effective method of conducting a Caries Risk Test, consistent with the findings of Liang and Xu et al. [14, 42]. Tanabe et al. [43] found satisfactory consistency in terms of outcomes between the CRT^®^ bacteria method and conventional methods of selective microbial culture and counting.

The CRT^®^ bacteria kit contains a special plate preprepared with MSB and Rogosa agar on different sides; thus, no special preparation is required; and it is characterized by its simple operation and measurement, with high reproducibility and feasibility, low technical requirements, ability to be used in large sample testing, and easy generalization [14, 42, 43]. However, this method requires incubation for 48 hours after sample collection and manual comparison of results rather than precise quantification. Therefore, the development of easy-to-use, fast, and accurate quantification methods would be a significant step forward for Caries Risk Testing.

## 5. Conclusions

The level of infection with oral SM and LB was positively correlated with caries status in children's primary teeth and the development and progression of caries. A high level of infection with oral SM and LB suggests a high prevalence of caries and predicts an increasing trend in the future, with a large number of decayed teeth and surfaces indicating more severe caries. Furthermore, infections with oral SM and LB are independent risk factors for caries in primary teeth, the risk of caries increasing approximately 10.9-fold when both salivary SM and LB counts >10^4^ CFU/mL. Finally, the CRT^®^ bacteria test is a facile yet effective form of the Caries Risk Test.

## Figures and Tables

**Table 1:** Caries status of 140 children of both genders over two years.

Examination	Gender	Number of participants	Number of caries cases	Caries prevalence (%)	*χ* ^2^	*P*	dmft ($\bar{x}\pm s$)	*Z*	*P*	dmfs ($\bar{x}\pm s$)	*Z*	*P*	CSI ($\bar{x}\pm s$)	*Z*	*P*
Initial exam	Boy	70	28	40.00	2.03	>0.05	1.46 ± 2.18	1.00	>0.05	2.07 ± 4.28	0.92	>0.05	4.23 ± 6.54	0.99	>0.05
	Girl	70	20	28.57			1.50 ± 2.91			2.39 ± 5.40			5.20 ± 11.14		
	Total	140	48	34.29			1.48 ± 2.56			2.23 ± 4.86			4.71 ± 9.11		

Follow-up exam after two years	Boy	70	46	65.71	0.03	>0.05	3.73 ± 4.11	−0.10	>0.05	5.93 ± 7.60	−0.10	>0.05	11.43 ± 14.19	−0.17	>0.05
	Girl	70	47	67.14			3.90 ± 4.39			6.23 ± 8.29			12.30 ± 15.82		
	Total	140	93	66.43			3.81 ± 4.24			6.08 ± 7.93			11.87 ± 14.98		

Increase over two years	Boy	70	18	25.71	2.65	>0.05	2.27 ± 2.83	−0.46	>0.05	3.86 ± 5.14	−0.39	>0.05	7.20 ± 9.88	−0.41	>0.05
	Girl	70	27	38.57			2.40 ± 2.79			3.84 ± 4.85			7.11 ± 8.55		
	Total	140	45	32.14			2.34 ± 2.80			3.85 ± 4.98			7.15 ± 9.20		

**Table 2:** Caries status of the 140 children in different CRT-SM levels over two years.

Examination	SM level	Number of participants	Number of caries cases	Caries prevalence (%)	SNK		*χ* ^2^	*P*	dmft ($\bar{x}\pm s$)	SNK		*χ* ^2^	*P*	dmfs ($\bar{x}\pm s$)	SNK		*χ* ^2^	*P*	CSI ($\bar{x}\pm s$)	SNK		*χ* ^2^	*P*
Initial exam	0	49	8	16.33	B		12.66	<0.001	0.45 ± 1.08	B		15.63	<0.01	0.53 ± 1.32	B		15.14	<0.01	1.22 ± 2.93	B		16.40	<0.001
	1	33	11	33.33	B	A			1.39 ± 2.50	B	A			2.15 ± 4.18	B	A			4.28 ± 9.67	B	A		
	2	31	15	48.39		A			2.19 ± 2.97		A			2.77 ± 4.43		A			6.45 ± 9.78		A		
	3	27	14	51.85		A			2.63 ± 3.33		A			4.78 ± 8.14		A			9.58 ± 12.30		A		

Follow-up exam after two years	0	49	25	51.02	B		11.07	<0.001	1.98 ± 2.76	C		23.71	<0.0001	2.82 ± 4.34	C		23.35	<0.0001	5.56 ± 8.49	C		24.69	<0.0001
	1	33	22	66.67	B				3.30 ± 3.87	C	B			5.27 ± 7.07	C	B			9.81 ± 13.39	C	B		
	2	31	22	70.97	B	A			4.52 ± 4.55		B			6.61 ± 7.44		B			13.83 ± 15.78		B		
	3	27	24	88.89		A			6.96 ± 4.69		A			12.37 ± 10.65		A			23.56 ± 18.20		A		

Increase over two years	0	49	17	34.69	A		0.06	>0.05	1.53 ± 2.27	B		14.74	<0.01	2.29 ± 3.83	B		19.03	<0.001	4.34 ± 7.42	B		17.93	<0.001
	1	33	11	33.33	A				1.91 ± 2.43	B				3.12 ± 4.23	B				5.53 ± 6.78	B			
	2	31	7	22.58	A				2.32 ± 2.59	B				3.84 ± 4.36	B				7.38 ± 8.11	B			
	3	27	10	37.04	A				4.33 ± 3.43	A				7.59 ± 6.45	A				13.98 ± 12.32	A			

*Note.* Differences between groups with identical letters denoting SNK ranking are not statistically significant, while differences between groups with different letters are statistically significant. The level of SNK is ranked alphabetically.

**Table 3:** Correlation between CRT-SM levels and caries status.

Indicators of caries status	SM level and indicators at the initial exam		SM level and indicators in the follow-up exam after two years		SM level and the increase in indicators over the two years	
	r	*P*	r	*P*	r	*P*
dmft	0.3323	<0.0001	0.4030	<0.0001	0.3047	0.0003
dmfs	0.3281		0.3983		0.3489	<0.0001
CSI	0.3426		0.4099		0.3444	

**Table 4:** Caries status of 140 children at the different CRT-LB levels over two years.

Examination	LB level	Number of participants	Number of caries cases	Caries prevalence (%)	SNK		*χ* ^2^	*P*	dmft ($\bar{x}\pm s$)	SNK		*χ* ^2^	*P*	dmfs ($\bar{x}\pm s$)	SNK		*χ* ^2^	*P*	CSI ($\bar{x}\pm s$)	SNK		*χ* ^2^	*P*
Initial exam	0	58	9	15.52	B		17.98	<0.0001	0.52 ± 1.35	B		21.58	<0.0001	0.67 ± 1.84	B		21.16	<0.0001	1.38 ± 3.60	B		21.97	<0.0001
	1	39	14	35.90	A				1.44 ± 2.52	B	A			1.85 ± 3.44	B	A			4.84 ± 9.98	B	A		
	2	27	16	59.26	A				2.70 ± 3.07		A			4.59 ± 6.78		A			8.75 ± 10.57		A		
	3	16	9	56.25	A				3.00 ± 3.56		A			4.81 ± 8.31		A			9.69 ± 13.26		A		

Follow-up exam after two years	0	58	32	55.17	B		7.97	<0.01	2.24 ± 2.96	B		20.83	<0.0001	3.31 ± 4.63	B		21.16	<0.0001	5.86 ± 8.30	B		24.08	<0.0001
	1	39	25	64.10	B	A			3.54 ± 4.42	B				5.41 ± 7.97	B				11.22 ± 15.98	B			
	2	27	23	85.19		A			6.56 ± 4.71	A				11.00 ± 9.52	A				21.99 ± 17.17	A			
	3	16	13	81.25	B	A			5.56 ± 4.29	A				9.44 ± 9.80	A				18.13 ± 17.11	A			

Increase over the two years	0	58	23	39.66	A		2.12	>0.05	1.72 ± 2.59	B		13.29	<0.01	2.64 ± 4.10	B		15.94	<0.01	4.48 ± 7.00	C		20.477	<0.0001
	1	39	11	28.21	A				2.10 ± 2.83	B				3.56 ± 5.61	B				6.38 ± 10.08	C	B		
	2	27	7	25.93	A				3.85 ± 2.96		A			6.41 ± 5.32		A			13.24 ± 9.94		A		
	3	16	4	25.00	A				2.56 ± 2.42	B	A			4.63 ± 4.32	B	A			8.44 ± 8.52	B	A		

Differences between groups with identical letters denoting SNK ranking are not statistically significant, while differences between groups with different letters are statistically significant. The level of SNK is ranked alphabetically.

**Table 5:** Correlation between CRT-LB levels and caries status.

Indicators of caries status	LB level and indicators at the initial exam		LB level and indicators in the follow-up exam after two years		LB level and the increase in indicators over the two years	
	r	*P*	r	*P*	r	*P*
dmft	0.3870		0.3598		0.2645	<0.01
dmfs	0.3804	<0.0001	0.3553	<0.0001	0.2931	<0.001
CSI	0.3892		0.3842		0.3243	<0.0001

**Table 6:** Single-factor logistic regression analysis of cariogenic bacterial infection.

Factors	Total cases	Caries cases	Caries-free cases	X^2^	*P*	*β*	OR	95% confidence interval
SM ≥ 10^4^ CFU/mL	91	40	51	10.79	<0.001	1.3911	4.019	1.695–9.530
SM <10^4^ CFU/mL	49	8	41					

LB ≥ 10^4^ CFU/mL	82	39	43	15.48	<0.0001	1.5969	4.938	2.148–11.352
LB < 10^4^ CFU/mL	58	9	49					

**Table 7:** Influence of cariogenic bacterial infection on caries status.

SM	LB	Caries cases (caries = 1)	Caries-free cases (caries = 0)	Total
SM ≥ 10^4^ CFU/mL(SM = 1)	LB ≥ 10^4^ CFU/mL (LB = 1)	35	29	64
	LB < 10^4^ CFU/mL (LB = 0)	5	22	27

SM <10^4^ CFU/mL(SM = 0)	LB ≥ 10^4^ CFU/mL (LB = 1)	4	14	18
	LB < 10^4^ CFU/mL (LB = 0)	4	27	31

**Table 8:** Multivariate logistic regression model for cariogenic bacterial infection.

Factors	Parameters	*χ* ^2^	*P*	OR	95% confidence interval
Intercept	−2.2740	23.00	<0.0001		
SM/*β*1	1.0442	5.08	<0.05	2.841	1.146–7.043
LB/*β*2	1.3482	9.40	<0.01	3.850	1.627–9.115

## Data Availability

The data used to support the findings of this study are restricted by the Ethics Committee of the Shenzhen Maternity and Child Healthcare Hospital Affiliated to Southern Medical University in order to protect children's privacy. The data that support the findings of this study are available from the corresponding author for researchers who meet the criteria for access to confidential data upon reasonable request.
